This article has been retracted.

# Sanitation, water, energy use, and traffic volume affect environmental quality: Go-for-green developmental policies

**DOI:** 10.1371/journal.pone.0271017

**Published:** 2022-08-26

**Authors:** Luqman Khalil, Shujaat Abbas, Kamil Hussain, Khalid Zaman, Iswan, Hailan Salamun, Zainudin Bin Hassan, Muhammad Khalid Anser

**Affiliations:** 1 Department of Economics, Government Post Graduate College No. 1, Abbottabad, KPK, Pakistan; 2 Graduate School of Economics and Management, Ural Federal University, Yekaterinburg, Russian Federation; 3 Department of Management Sciences, University of Wah, Wah Cantt, Pakistan; 4 Department of Economics, The University of Haripur, Haripur, Khyber Pakhtunkhwa, Pakistan; 5 Education Faculty, University of Muhammadiyah Jakarta, South Jakarta, Indonesia; 6 Department of Nationhood and Civilization, Centre for Fundamental and Continuing Studies (PPAL), Universiti Malaysia Terengganu (UMT), Kuala Nerus, Terengganu, Malaysia; 7 School of Education, Faculty of Social Sciences and Humanities, Universiti Teknologi Malaysia (UTM), Skudai, Johor Bahru, Malaysia; 8 School of Public Administration, Xi’an University of Architecture and Technology, Xi’an, China; 9 Faculty of Business and Management Sciences, The Superior University, Lahore, Pakistan; Northeastern University (Shenyang China), CHINA

## Abstract

Carbon emissions are primarily the result of human activity in urban areas. Inadequate sanitary facilities, contaminated drinking water, nonrenewable energy, and high traffic congestion have all impacted the natural ecosystem. Using data from 1975 to 2019, the study assessed the impact of the aforementioned variables on Pakistan’s carbon emissions in light of this crucial fact. The ARDL cointegration method was used to estimate the short- and long-run parameter estimates. Urban sanitation challenges and energy consumption increase carbon emissions, which affects the natural environment by raising a country’s carbon intensity. Economic expansion confirmed the inverted U-shaped relationship between carbon emissions and economic growth to verify the Environmental Kuznets Curve (EKC) hypothesis in the long run. In contrast, the monotonically rising function of carbon emissions provides evidence of the nation’s economic development in the short run. Access to clean drinking water improves population health and encourages the purchase of eco-friendly products. The government must improve sanitation services and use renewable energy sources to enhance air quality.

## 1. Introduction

The continuation of hygienic conditions in urban areas is linked to urban sanitation, and city sanitation is a far more intricate system [1]. Cleanliness is a recurring issue in slums, as crowded conditions and a lack of cleanliness lead to disease outbreaks that imperil shantytown inhabitants while exposing other city residents to health risks [2]. The goals of urban sanitation are to reduce the risk to human health by addressing the factors that might cause health issues [3]. Poor sanitation is linked to the spread of illnesses that harm public health. The United Nations General Assembly recognized uncontaminated drinking water and hygiene as fundamental human rights in 2010 and called for worldwide efforts to help nations provide safe, fresh, controllable, and acceptable drinking water and cleanliness [4]. Target 6.2 of the Sustainable Development Goals calls for adequate and safe sanitation for all [5]. According to WHO [6] research, over 830,000 people die each year in low- and middle-income countries due to a faulty hygiene system, accounting for more than 60% of all diarrheal deaths. In addition, only 45 percent of the population used basic sanitation in 2017, and 2.2 billion people lacked access to non-toxic drinking water. Almost 4 billion people do not have a safe location to use a toilet.

Pakistan met the MDG for sanitation in 2015, lowering the proportion of people who lack balanced access to basic hygiene by half. Growing access to sanitation in rural areas accounts for 67 percent of the total in 2019, more than three times in 1991. As a result, about one-fourth of individuals in communities practice open defecation. Almost no money has been spent on mud or wastewater management. In rural Punjab, 42 percent of houses lack a drainage system, while 60 percent in rural KP lack one. In rural Punjab and KP, 1% and 10% have decent sanitation infrastructure. Sewer-connected toilets are available to more than 40% of urban KPK residents and almost 60% of urban Punjab residents. The relationship between toilets and sanitation is an essential indicator of safety measures [7, 8]. The availability of water, sanitation, and cleaning amenities vary between and within the KPK and Punjab areas. Approximately 90% and 85% of the populace now have safer water supplies and sanitation services, respectively [9]. Similarly, 94 percent of people have improved water sources in the Punjab region, and 72 percent have improved sanitation facilities [10]. There are significant differences between urban and rural regions at the district level within provinces. In 2015, UNICEF said that disparities should be reduced to achieve global sanitation [11].

As the complexity of contemporary living increased, so did energy usage. The notion of smart cities as creative hubs cannot be imagined without substantial use of various types of energy [12–14]. The need for energy is a crucial fuel for contemporary economies to function. EUSE is required for the operation of our companies, the lighting of our streets, and the powering of our automobiles [15, 16]. The combination of industrial growth and population growth has led to an unprecedented increase in energy use [17, 18]. Countries are working to keep the energy supply stable. The scarcity of energy has hampered economic development and lowered living standards [19–21]. Energy use is directly proportional to CO2 emissions. Since Rachel Carson’s book "Silent Spring" in 1962, which examines the consequences of biological variety, ecological concerns have gained prominence [22].

ICT penetration has expanded in underdeveloped countries, yet infrastructure and affordability are lacking. To stimulate ICT infrastructure investment, create and deploy modern information systems, leverage the financial sector to finance ICT projects at a reasonable interest rate, and encourage community demand on politicians to minimize unsustainable practices through strengthening e-government infrastructure [23].Today, one of the most significant global issues is attempting to bring the carbon pollution linked to increasing temperatures under control. To correctly manage economic and environmental resources, it is necessary to have a solid understanding of governance processes that consider the interconnected nature of environmental, social, and governance issues [24]. Countries should strengthen energy collaboration and consolidate national energy activities by balancing the critical components of the global energy paradox to aid in developing a well-balanced energy system [25]. Energy generation contributes to the ongoing easing of suffering and recommends feed-in pricing, tax credits, and the diversification of energy resources away from fossil fuels and toward renewable power sources [26]. The lack of available energy increases environmental stress. However, the advancement of education had a significant effect on sustainable development that contributed to globalization [27].

The generally accepted EKC theory links economic growth and environmental deprivation [28–30]. The notion of EKC emerged in the early 1990s due to Grossman and Krueger’s pioneering work and the World Bank’s development report [31]. Economic growth and ecological security are dynamically linked by an intertemporal restriction caused by the negative impact of pollutants on production. The EKC Hypothesis, which establishes an inverted U-shaped relationship between production and ecological quality, finds a significant correlation between environmental deterioration and growth in economic activity [32, 33]. Economic growth causes environmental degradation in low-income countries, but it reduces environmental impact in technologically advanced countries [34–36]. The link between energy use and increased economic interest concerns energy consumption and ecological issues [37] since environmental pollution is a severe issue caused by traditional energy sources. To a certain extent, conventional energy usage can disclose the current state of local environmental stress. Industrial actions substantially increased traffic and mono-nitrogen oxide (NOx) emissions across states. Trade volume, energy use, and food variability per capita are all tied to air pollutants that degrade the natural environment [38–40].

Based on the discussions, the study offered a series of research questions to be addressed in order to derive certain policy conclusions, first, whether insufficient urban sanitation causes a country’s high carbon intensity? The question is critical for analyzing the country’s sanitary infrastructure, which leads to the country’s environmental requirements. The second question is whether access to clean drinking water helps to enhance healthcare facilities, hence reducing environmental problems? The question was about contaminated and unsanitary drinking water, which caused many ailments, weakened the immune system and was most likely caused by environmental pollution. As a result, having access to safe drinking water is beneficial in resolving healthcare concerns and related environmental dangers in a country. Finally, does sustained economic expansion, nonrenewable energy fuels, and high traffic volume raise the cost of a country’s carbon emissions? The matter is critical since significant carbon emissions from the country’s commercial projects feed economic activity with nonrenewable fuels and high traffic volume. To lessen the negative impact of environmental externalities on the country, it is critical to move toward sustainable development projects paired with green energy sources and electric automobiles. The study presented the following research objectives in line with the research questions:

- To look at how urban sanitation, clean drinking water, and energy use affect carbon emissions in a country.
- To determine how high-volume traffic affects carbon emissions in a country when the EKC hypothesis is in place.
- To investigate the function of continued economic growth in reducing carbon emissions.

It helps make long-term policy suggestions when the results are compared with the goals. Various statistical tools are used to do this.

The significance of the research lies in its contribution to developing a resilient metropolitan system supported by clean drinking water, hygienic conditions, and a sustainable transportation system. Pakistan’s economy is supported by abundant valuable environmental and natural resources, which contribute to the country’s economic prosperity. However, the nation faced various additional difficulties relating to clean drinking water and urban sanitation services, which directly impacted the sustainability agenda for healthcare. In addition, increased energy use and transportation emissions threaten the green development goal, which requires a sustainable policy mix. Based on the issue, the study evaluated the given concerns and proposed sound policy inferences to improve the country’s natural environment and pave the way for green development.

## 2. Literature review

The massive increase in carbon output levels has prompted authorities to develop green and clean energy regulations. The prior research mainly examined several variables that reduce carbon emissions to pre-industrial levels [41, 42]. However, the ambition of reducing carbon emissions is still a long way from being a reality. The significant rural-urban migration places an immense strain on urban sanitation infrastructure, impacting the physical environment. The increased carbon emissions were exacerbated by inadequate sanitary facilities, resulting in increased healthcare costs. Willcock et al. [43] investigated the value of nature’s sanitation services. Human waste is channeled through nature and treated by plants, and nature cleanses over 42 million tonnes of human waste each year, a USD 4.4 billion services. Using data from 1972 to 2014, Ali et al. [44] investigated the relationship between CO2 emissions and urbanization in Pakistan. They discovered that urbanization increases CO2 emissions in both the long and short term. The increased requirement for urban planning and infrastructure development is critical to reducing a country’s negative environmental consequences. From 1970 to 2015, Liu and Bae [45] investigated the impact of industrial expansion and urban sprawl on carbon emissions in China. They discovered a substantial, long-term relationship between the alleged elements. Bekhet and Othman [46] discovered that early phases of urbanization (URB) had a detrimental influence on Malaysia’s environmental quality; however, it improves as the game progresses. Dogan and Turkekul [47] investigated the relationship between CO2 emissions, real GDP, energy use, free trade, urbanization, and financial development in the United States from 1960 to 2010. The study’s findings indicated that urbanization reduced green value in the long run, but two-way causal relationships were discovered in the short run. The other aspects must be carefully considered during policy proposals. Tyagi et al. [48] researched the causes and implications of environmental degradation. They discovered that minimizing exposure to environmental risk concerns increases air quality and offers better-quality drinking and cleaning water and sanitation sources. Clean energy has been linked to several health advantages. It is determined to make a significant contribution to the Millennium Development Goals. The link between urbanization and CO2 emissions in MENA economies was studied by Al-Mulali et al. [49]. The study’s outcomes suggest that urbanization positively impacts energy consumption and CO2 emissions. They claimed that urbanization increased energy use, especially fossil fuels, resulting in pollution.

Researchers investigating the link between energy use and economic development came with contradictory findings. Kraft and Kraft [50] demonstrated a one-way causality between energy usage and GDP and validated the conservation hypothesis using the years 1947–1974. According to the findings, energy usage significantly influences a country’s growth. Soytas and Sari [51] used data from 1950 to 1992 to support the conservation hypothesis in Japan, Germany, Turkey, and France, implying that economic expansion leads to massive energy consumption. The Argentineans verified the energy usage and production feedback, and Italy and Korea adopted the growth concept. Streimikiene and Kasperowicz [52] validated the energy-led growth postulate in a panel of 18 nations to support green growth initiatives. Gorus and Aydin [53] examined the relationship between energy usage, economic development, and CO2 emissions in MENA countries using panel data from 1975 to 2014. The findings indicate that energy management strategies boost economic growth, but their long-term repercussions are the opposite. Furthermore, no relationship exists between economic growth and carbon emissions. Legislators can enact CO2 emission controls and other ways to reduce pollution in the atmosphere. Using data from 249 Chinese cities in 2015, Xie et al. [54] evaluated if the EKC hypothesis holds between economic growth and pollution in China. The study employed a nonlinear spatial autoregressive model for the investigation. The results showed that PM2.5 pollutants have significant positive geographical spillover characteristics. They suggested that local governments modify the industrial structure to accommodate lower-income cities and encourage green industries. Zhang et al. [55] analyzed carbon emissions from Chinese transportation. The economic, technological, and managerial elements of traffic flow have been investigated, and they noticed that CO2 emissions computed using different approaches varied. As a result, it is critical to concentrate on dependable estimating methodologies. Mikayilov et al. [56] investigated the link between economic growth and carbon emissions in Azerbaijan from 1992 to 2013. The findings reveal that economic growth and CO2 emissions are positively connected in the long term. They suggest that carbon pricing tools and public awareness campaigns may be implemented to mitigate the adverse effects of pollution. Faridi and Murtaza [57] demonstrated a relationship between disaggregated economic development, energy consumption, and agricultural value-added in Pakistan. The country’s reliance on energy and gas means consumption increases faster than supply, which hurts output and exports. Secondary data from 1972 to 2011 was used in the study. According to the research, energy consumption and gas utilization are critical elements in increasing agricultural productivity and development. They also found that disaggregated energy use, economic growth, and agricultural production are linked to long-term growth.

Some of the recent publications on urban sanitation and carbon emissions are Li et al. [58], Chen et al. [59], Ortz-Rodriguez et al. [60], Zhang et al. [61], and Collaço & da Curz [62]. Due to unsanitary circumstances, these studies mostly restricted the carbon footprint, worsening the natural environment. Zakari et al. [63] suggested that it is possible to acquire environmentally friendly technology to reduce harmful emissions. Nevertheless, the authorities should create and implement rules against power generation systems that are not eco-friendly and have the potential to harm the environment. Following the debate, the following hypothesis was developed: Khan et al. [64] concluded that the sustainability of the ecosystem declines when natural resources are used up. Clean energy contributes to an increase in environmental quality and a slowing of economic growth. Both energy security and ecological sustainability benefit from the transition to renewable energy. Khan et al. [65] further argued that governments should embrace sustainable tax changes to overcome worldwide environmental concerns and achieve a greener future. Government spending should be linked with environmental goals, pricing should reflect externalities, and fiscal reform should allow for green environment investment to achieve sustainable development goals. Zakari et al. [66] suggested that when there are specialized institutional procedures and energy sources, there is the possibility of improving the ecological footprint.

***H1*: *If there is not enough sanitation in cities*, *more natural distortions will happen*, *which will lead to more carbon emissions in a country*.**

The stated hypothesis examines a country’s existing urban sanitation position about the environmental sustainability agenda or the blue economy. Furthermore, the present literature favors adequate access to safe drinking water to promote healthy hygiene. It prefers to use eco-friendly items that increase environmental quality levels [67–71]. Based on the issue’s significance, the study developed the second hypothesis,

***H2*: *Uncontaminated drinking water is likely to attain healthcare sustainability in a country*.**

Finally, there is a plethora of work on the EKC hypothesis, energy-related emissions, and transportation emissions in various economic situations, for example, Erdogan et al. [72], Amin et al. [73], Shikwambana et al. [74], Murshed et al. [75], and Alola et al. [76]. According to these studies, the environmental sustainability agenda might be achieved by utilizing sustainable transportation, green energy consumption and production, and green development initiatives. The following is the hypothesis of the study, i.e.,

***H3*: *Continued economic expansion*, *nonrenewable fuels*, *and high traffic intensity are all expected to raise the cost of a country’s carbon emissions*.**

The real contribution of the research is to integrate several sustainable aspects into the resource conservation agenda, paving the way for global prosperity. First, the research investigates the effect of urban sanitation on the natural environment in densely populated places. The prior studies evaluated the indirect cost of sanitary infrastructure on environmental degradation while discounting the intensity of traffic loads, which is directly connected to the green development approach [77–79]. Second, the research included safe, non-polluted drinking water, which contributes to the improvement of public health and the promotion of a green and clean environment. Prior research supports the supplied assertion; however, just a few studies have examined the relationship between emissions and income [80–82]. The research used energy consumption as a reference for the emissions-income-sanitation nexus, which assists in evaluating urban infrastructure and energy sources to reduce carbon abatement costs. Prior studies focused on energy consumption and carbon emissions but little investigate other aspects that may have been significant; thus, these factors are crucial for investigation for long-term sustainable growth [83–85].

## 3. Data sources and methodological framework

The study analyzed data from 1975 to 2019 to examine CO2 emissions, urban sanitation, urban access to clean drinking water, energy consumption, traffic volume, and economic growth in Pakistan. The World Bank [86] provided the statistics for the criteria above. The variables are listed in Table 1.

**Table 1:** List of variables.

Variables	Symbol	Measurement	Definition
Carbon dioxide emissions	CO2	kiloton	CO2 emissions are produced when fossil fuels are burned. Solid, liquid, and gaseous fuels are used to make it.
Urban sanitation	USAN	% of urban population	The proportion of city dwellers who use sanitation services and have them securely handled. Latrines and flushing to piped sewer systems are also incorporated.
Urban access to safe drinking water	UASDW	% of urban population	The proportion of total urban residents who get their drinking water from a higher-quality source with a round-trip delivery time of less than half an hour. Better-quality sources include tube wells, hand pumps, and line pipes.
Gross domestic product	INCOME	Current US$	Throughout the fiscal year, the market value of currently generated products and services offered by all citizens of the country.
Energy use	EUSE	kg of oil equivalent per capita	It refers to the use of primary energy prior to its conversion to other end-use fuels.
Traffic volume	TVOL	TEU: 20-foot equivalent units	The container port traffic statistics assess the volume of traffic intensity.

The study started with the Solow growth model [87], which established the foundation for current economic theory. The Solow Growth model is an exogenous model that analyses variations in an economy’s output levels over time due to population fluctuations. The production function determines the source of goods, which asserts that production is determined by the stock of capital and labor force, i.e.,

Y=F(K,L) (1)

The Solow model employs the constant return to scale (CSR) hypothesis for the production function. This is a valid assumption. It makes the analysis easier. If the output function has a CSR, then

zY=F(zK,zL) (2)

Assume z is a positive number. When ’z’ is multiplied by both capital and labor, the quantity of output is also multiplied by z. We may investigate all quantities in the economy concerning the size of the labor force using production functions and CSR. The study, which was based on the Solow growth model, replaced economic growth of its byproduct, i.e., carbon emissions, which are generated during economic output, i.e.,

$$CO2=\beta_{0}+\beta_{1}USAN+\beta_{2}UASDW+\beta_{3}INCOME+\beta_{4}{\left(INCOME\right)}^{2}+\beta_{5}EUSE+\beta_{6}TVOL+\varepsilon$$ (3)

Fig 1 shows the trend analysis of the variables for ready reference. Carbon emissions persistently increases due to an increase in energy use, continued economic growth, traffic volume, and unhygienic basic sanitation services over a time period.

**Fig 1:** Trend analysis of the studied variables. Source: World Bank [86].

The ARDL bounds test, introduced by Pesaran et al. [88], was used in this study to determine the long-term relationship between the mentioned variables. ARDL provides several benefits over Johanson Cointegration and other approaches, ass described by Pesaran et al. [89], i.e.,

- In an ARDL estimation, all variables in the same order may or may not be stationary.
- The ARDL method yields reliable results in finite samples; and
- The ARDL application delivers unbiased long-run model estimates by combining integrated variables in a single regression apparatus [90].

The following is the ARDL specification:

$$\begin{array}{l} \Delta \mathrm{CO}2=\alpha_{o}+\alpha_{1}\mathrm{CO}2_{t‐1}+\alpha_{2}{\mathrm{EUSE}}_{t‐1}+\alpha_{3}{\mathrm{USAN}}_{t‐1}+\alpha_{4}{\mathrm{UASDW}}_{t‐1}+\alpha_{5}{\mathrm{TVOL}}_{t‐1}+\alpha_{6}{\mathrm{INCOME}}_{t‐1}+\\ \alpha_{7}{\mathrm{INCOME}}^{2}{}_{t‐1}+\overset{k}{\underset{i=0}{\sum }}\alpha_{i}\Delta \mathrm{CO}2+\overset{m}{\underset{j=0}{\sum }}\alpha_{j}\Delta \mathrm{EUSE}+\overset{o}{\underset{k=0}{\sum }}\alpha_{k}\Delta \mathrm{USAN}+\overset{p}{\underset{l=0}{\sum }}\alpha_{1}\Delta \mathrm{UASDW}+\\ \overset{Q}{\underset{m=0}{\sum }}\alpha_{m}\Delta \mathrm{TVOL}+\overset{R}{\underset{n=0}{\sum }}\alpha_{n}\Delta \mathrm{INCOME}++\overset{R}{\underset{n=0}{\sum }}\alpha_{n}\Delta {\mathrm{INCOME}}^{2}+e_{i} \end{array}$$ (4)

Where; Δ is the first difference of the variables.

The error correction term (*p*) shows the adjustment of the stated variables towards the long-run equilibrium; hence it is included in Eq (4) for robust inferences, i.e.,

$$\begin{array}{l} \Delta \mathrm{CO}2=\alpha_{o}+\alpha_{1}\mathrm{CO}2_{t‐1}+\alpha_{2}{\mathrm{EUSE}}_{t‐1}+\alpha_{3}{\mathrm{USAN}}_{t‐1}+\alpha_{4}{\mathrm{UASDW}}_{t‐1}+\alpha_{5}{\mathrm{TVOL}}_{t‐1}+\alpha_{6}INCOME_{t‐1}+\\ \alpha_{7}{\mathrm{INCOME}}^{2}{}_{t‐1}+\overset{k}{\underset{i=0}{\sum }}\alpha_{i}\Delta \mathrm{CO}2+\overset{m}{\underset{i=0}{\sum }}\alpha_{j}\Delta \mathrm{EUSE}+\overset{o}{\underset{k=0}{\sum }}\alpha_{k}\Delta \mathrm{USAN}+\overset{p}{\underset{l=0}{\sum }}\alpha_{1}\Delta \mathrm{UASDW}+\\ \overset{Q}{\underset{m=0}{\sum }}\alpha_{m}\Delta \mathrm{TVOL}+\overset{R}{\underset{n=0}{\sum }}\alpha_{n}\Delta \mathrm{INCOME}++\overset{R}{\underset{n=0}{\sum }}\alpha_{n}\Delta {\mathrm{INCOME}}^{2}+p+e_{i} \end{array}$$ (5)

The null hypothesis of no cointegration would be assessed through Wald F-statistics, i.e.,

H0: α_1_ = α_2_ = α_3_ = α_4_ = α_5_ = α_6_ = α_7_ = 0
H1: α_1_ ҂ α_2_ ҂α_3_ ҂ α_4_ ҂α_5_ ҂ α_6_ ҂α_7_ ҂0

The Narayan critical values of I(0) and I(1) bound values are assessed for the cointegration process.

## 4. Results and discussion

The descriptive statistics for the variables are shown in Table 2. Carbon emissions have a low value of 331.783 and a high value of 987.832, with an average value of 700.061. The variable has a skewed distribution, with a standard deviation of 211.862. The average value of energy consumption, income, and traffic volume is around 413.699 kg of oil equivalent per capita, 815.350 US dollars, and 1404729 traffic intensity. The average value of urban sanitation and access to clean drinking water in cities is 68.220 percent and 94.898 percent of the total urban population. Traffic volume has a high peak of distribution, followed by urban sanitation, GDP, safe drinking water, energy use, and carbon emissions.

**Table 2:** Descriptive statistics.

Methods	CO2	EUSE	INCOME	TVOL	UASDW	USAN
Mean	700.061	413.699	815.350	1404729	94.898	68.220
Maximum	987.832	500.432	1197.913	3460700	95.149	76.619
Minimum	331.783	299.104	477.967	878892	94.224	65.688
Std. Dev.	211.862	61.047	199.867	804428.4	0.334	3.861
Skewness	-0.241	-0.623	0.070	1.230	-0.876	1.218
Kurtosis	1.728	1.974	2.600	3.203	2.221	2.892

Table 3 illustrates that energy consumption, national income, traffic volume, and urban cleanliness all positively correlate with carbon emissions. In contrast, access to safe drinking water in cities is adversely associated with carbon emissions. Income, traffic volume, and urban cleanliness, on the other hand, raise a country’s energy consumption, and the amount of traffic was shown to be positively connected with the country’s income. The findings revealed that ongoing economic expansion, energy usage, traffic intensity, and insufficient sanitation facilities are natural environmental variables that worsen carbon emissions in a nation. To move forward with the green development strategy, the country should adopt strict economic measures.

**Table 3:** Correlation matrix.

Variables	CO2	EUSE	INCOME	INCOME^2^	TVOL	UASDW	USAN
CO2	1						
EUSE	0.958***	1					
INCOME	0.982***	0.905***	1				
INCOME^2^	0.958***	0.852***	0.992***	1			
TVOL	0.779***	0.584***	0.855***	0.910***	1		
UASDW	-0.833***	-0.657***	-0.884***	-0.926***	-0.969***	1	
USAN	0.772***	0.568***	0.846***	0.897***	0.982***	-0.978***	1

Note

*** indicates 1% significance level.

Time-series data necessitates the investigation of data stationarity as a first step. As shown in Table 4, the analysis variables were not integrated into the same sequence. The findings indicate that CO2 emissions, uncontaminated clean drinking water, and urban sanitation are stationary variables. Energy consumption, income, and traffic volume, on the other hand, differ in a stationary manner. So, because of this, the ARDL Bounds testing method can be used to ensure that the results are reliable.

**Table 4:** ADF unit root estimates.

Variables	Level			First Difference			Order of Integration
	None	Intercept	both	None	Intercept	Both	
CO2	8.132	-4.638***	-------	---------	-----------	-----	I(0)
EUSE	3.267	-2.455	0.014	-4.212***	-----------	----	I(1)
INCOME	6.186	-1.804	-2.610	-1.656*	-5.500***	------	I(1)
TVOL	1.528	0.261	-1.575	-3.692***	--------	------	I(1)
UASDW	-3.710***	------	-------	-------	-------	-------	I(0)
USAN	0.5937	-3.822***	-------	--------	------	-------	I(0)

Note

*** and * indicates 1% and 10% level of significance.

The ARDL Bounds testing estimates and Variance Inflation factor (VIF) for detecting multicollinearity are shown in Table 5. The reported Wald F-statistics value is 8.272, greater than the upper bound critical value of 1% significance. As a result, we could be sure that the cointegrated process matched up with the variables in the shown model. Further, the VIF value is less than the value of 10, hence, the study safely conclude the absence of multicollinearity in a given model.

**Table 5:** ARDL bounds test estimates.

Test Statistics	Value	Degree of freedom	Variables	VIF
F-statistics	8.272	6	Constant	NA
**Significance Level**	**I(0)**	**I(1)**	Δln(EU)	1.370
10%	1.75	2.87	Δln(GDP)	1.102
5%	2.04	3.24	Δln(TRAFFIC)	1.391
2.5%	2.32	3.59	Δln(UASDW)	1.725
1%	2.66	4.05	Δln(USAN)	2.074

The short-run ARDL estimations are shown in Table 6. The findings indicate that urban sanitation infrastructure is insufficient to reduce carbon emissions. It is critical to enhancing urban hygiene to avoid negative environmental externalities that impede the country’s long-term efforts [91–93]. By achieving public health, access to clean and sterilized safe drinking water significantly reduces the cost of carbon emissions. Water treatment, the provision of clean and purified water, the chlorinated drinking water system, and ultrafiltration are just a few examples of sustainable water solutions that improve general public health and achieve healthcare sustainability [94–96]. As sustained economic expansion jeopardizes environmental damage in the form of growing carbon emissions, the country’s GDP follows the monotonic increasing function of carbon emissions. If a country’s carbon emissions are too high, it could use strict environmental policies [97], incentive-based regulations [98], and carbon pricing [99] in the long term.

**Table 6:** ARDL short-run estimates.

Variables	Coefficients	S. Error	t-statistics	Probability
D(USAN)	10.007	3.241	3.087	0.003
D(UASDW)	-11.775	2.438	-4.828	0.000
D(TVOL)	0.000012	0.00002	0.596	0.554
D(EUSE)	1.845	0.273	6.738	0.000
D(INCOME)	0.505	0.258	1.954	0.058
D(INCOME)^2^	-0.00019	0.00015	-1.206	0.235
CointEq(-1)	-0.889	0.097	-9.141	0.000

Note: Dependent variable: D (CO2). CointEq(-1) shows error correction term.

Table 7 displays the ARDL long-run estimations, which verified the EKC hypothesis with a turning point of US$ 729. Haans et al. [100] suggested a way to analyze EKC and get estimate itsturning point, which followed in the given study and confirmed the inverted U-shaped relationship between the country’s economic growth and carbon emissions. Energy consumption positively correlates with carbon emissions, which validates energy-embodied products. Carbon excretions are positively and negatively associated with urban sanitation systems and clean drinking water, and the latter validated the higher carbon emissions caused by insufficient urban sanitation services. On the other hand, the former underlined the importance of clean drinking water in improving public health hygiene elements and accomplishing the healthcare sustainability target. Several previous investigations, including Sarkodie and Ozturk [101], Murshed et al. [102], Erdogan et al. [103], and Suki et al. [104], corroborated the EKC theory by energy embodied emissions. These investigations confirmed that energy fuels hinder the green development strategy. Alternative power energies should be used to meet energy efficiency and other goals [105–107].

**Table 7:** ARDL long-run estimates.

Variables	Coefficients	S. Error	t-Stat.	Probability
INCOME	0.001458	0.000626	2.330607	0.0253
INCOME^2^	-0.000001	0.0000004794	-2.085844	0.0439
**EKC Turning Point = -(INCOME/2˟INCOME** ^**2**^ **) = US$729**				
EUSE	2.384174	0.476289	5.005727	0.0000
TVOL	-0.152837	0.106540	-1.434559	0.1598
UASDW	-4.199069	1.187151	-3.537097	0.0011
USAN	3.944168	1.097968	3.592245	0.0009
**Diagnostic Testing**				
J.B Test	1.104 (0.575)	Heteroskedasticity Test		1.051 (0.418)
Autocorrelation LM Test	1.223 (0.307)			
Ramsey RESET Test	1.653 (0.106)			

Note: small bracket shows probability value.

Furthermore, urban sanitation increases carbon emissions, yet urban access to clean drinking water improves health hygienic aspects, resulting in healthcare sustainability. Previous research corroborated the study’s findings by identifying many sustainable elements that contribute to good sanitation services and the supply of clean drinking water. For example, Dickin et al. [78] underlined the need to improve sanitation services through climate finance sources that aid in achieving long-term cleanliness. Anser et al. [108] stated that urbanization and sustained economic expansion are the primary causes of rising carbon emissions, and both must be addressed through urban planning and incentive-based legislation. Li et al. [58] said that decentralizing water treatment through new technology that makes drinking water safe and clean was important. The diagnostic test estimates confirmed the absence of normality issue, serial correlation, heteroskedasticity, and measurement issue in the given model.

The CUSUM test verifies the model’s parameter stability. To understand the findings, the order of sums and squares of recursive residuals is determined from subsamples of the data. The null hypothesis of parameter constancy states that the model is unstable or that structure change occurs over time based on the sequence values outside of the model. The alternative hypothesis confirms that the model is stable and the values remain within the residual series. Fig 2 depicts the CUSUM and CUSUM square statistics, revealing that the model is stable over time and statistically significant at a 5% significance level.

**Fig 2:** CUSUM and CUSUM square estimates. Source: Author’s estimates.

## 5. Conclusions and policy recommendations

The study’s purpose is to assess the three primary United Nations objectives, including SDG-6, SDG-7, and SDG-13, in the context of Pakistan. Pakistan’s economy was confronted with health-related challenges, including polluted drinking water and increased carbon emissions. The study assessed the parameters mentioned above by gathering data from 1975 to 2019 using the ARDL Bounds testing technique. The results validate the EKC hypothesis in the long run, but the connection between the two elements becomes a monotonic growing function in the short run. The urban sanitation system is ineffective in mitigating the adverse effects of environmental externalities while exacerbating carbon emissions. Fresh and safe water intake enhances ordinary people’s health hygiene and proclivity to buy eco-friendly items to minimize carbon emissions. Because of the substantial usage of energy fuels in the whole energy mix, energy demand raises carbon emissions. The study provided the following strategic plans based on the stated results:

- The issue of sanitation highlights the need for a broader perspective on adaptation, one that considers the challenge of providing equal access to essential services for the world’s poorest populations while also adjusting to the dangers posed by climate change. To improve climate finance for sanitation projects, investors need to know better about this relationship, especially about initiatives that promote equitable access via flexible and low-emission technologies.
- Access to safe and uncontaminated drinking water is another critical component of the healthcare sustainability agenda. Water-borne infections are disseminated mainly by contaminated and filthy drinking water, posing serious health risks. Public labs should clean the water and put up public water filters so people can get clean and clear drinking water quickly.
- The travel and transportation systems should be electrified and run on renewable energy fuels to prevent carbon emissions. The level of traffic should be managed, and sustainable ways of public transit should be used. The government should charge very little for public transportation, which helps cut down on carbon emissions by cutting down on traffic.
- The greater reliance on fossil fuel combustion for economic enterprises must be replaced by renewable fuels, resulting in carbon neutrality. Exploring the plentiful renewable energy resources for energy production is critical for policymakers to uncover the stock of biomass energy and biogas, which are less sensitive to the environment, and
- Continued economic expansion necessitates greater emissions to complete the life cycle of their manufacturing process. As a result, the cost of carbon emissions has risen, having a significant impact on green and clean development goals. The few critical policy components supporting economic growth while reducing carbon emissions are incentive-based environmental legislation, strong command-and-control mechanisms, carbon pricing, green energy utilization, and technical innovation.

The five-point plan would help us be more energy-efficient and solve long-term water and sanitation problems so that we can move forward toward a healthier future.
